RETRACTED

# LncRNA HCG11 regulates proliferation and apoptosis of vascular smooth muscle cell through targeting miR-144-3p/FOXF1 axis in atherosclerosis

**DOI:** 10.1186/s40659-020-00306-2

**Published:** 2020-10-02

**Authors:** Yi Liu, Xiyun Cui, Cong Wang, Sihai Zhao

**Affiliations:** 1 Department of Clinical laboratory, The First Affiliated Hospital of Xi’an Jiaotong University, Xi’an, Shaanxi 710061 China; 2 Department of Clinical Laboratory, Weapon Industry 206 Hospital, Xi’an, Shaanxi 710061 China; 3 Laboratory Animal Center, Xi’an Jiaotong University School of Medicine, Xi’an, Shaanxi 710061 China

**Keywords:** LncRNA HCG11, MiR-144-3p, FOXF1, Cell proliferation, Apoptosis, Atherosclerosis

## Abstract

**Background:**

Atherosclerosis (AS) is the main pathological basis of coronary heart disease, cerebral infarction and peripheral vascular disease, which seriously endanger people’s life and health. In recent years, long non-coding RNA (lncRNA) has been found to be involved in gene expression regulation, but the research on AS is still in the initial stage. In this study, we mainly studied the role of HCG11 in patients with AS. Quantitative Real-time Polymerase Chain Reaction (QRT-PCR) was used to detect the expression of HCG11 and miR-144 in the serum of AS patients and healthy volunteers. Oxidation Low Lipoprotein (Ox-LDL), interleukin-6 (IL-6) and tumor necrosis factor α (TNF α) radiation were used to establish human vascular smooth muscle cells (VSMCs) in vitro model. Cell proliferation was determined by Cell Counting Kit-8 (CCK-8) assay. The apoptosis rate was determined by flow cytometry (FACS) and terminal deoxynucleotidyl transferase-mediated dUTP-biotin nick end labeling assay (TUNEL) staining. The expression levels of Forkhead box protein F1 (FOXF1), B cell lymphoma-2 (Bcl-2) and BCL2-Associated X (Bax) were detected by qRT-PCR. Luciferase gene reporter and RNA pull down experiments confirmed the relationship between HCG11 and miR-144, miR-144 and FOXF1.

**Results:**

This study showed that HCG11 was significantly upregulated in patients with AS, while miR-144 was down-regulated in patients with AS. Ox-LDL and IL-6 in VSMCs induced up-regulation of HCG11 and down-regulation of miR-144. Overexpression of HCG11 promoted the proliferation and inhibited apoptosis of VSMCs. Luciferase gene reporter gene assay showed that HCG11 could bind to miR-144, and miR-144 could bind to FOXF1. Overexpression of miR-144 reversed the effect of HCG11 on VSMCs.

**Conclusions:**

LncRNA HCG11 regulates proliferation and apoptosis of vascular smooth muscle cell through targeting miR-144-3p/FOXF1 axis.

## Background

The development of atherosclerosis is a complex process involving the interaction of various cells and cytokines [1–3]. A variety of cells are involved in the development of atherosclerosis, including lymphocytes, macrophages, endothelial cells, and smooth muscle cells (SMCs). Histological studies of human coronary arteries suggest that areas prone to atherosclerotic lesions contain more vascular SMCs, while areas less prone to atherosclerotic lesions have fewer vascular SMCs [4–6]. Therefore, understanding the relationship between VSMCs and AS may have important implications for the formulation of effective prevention and control measures for AS [7–9].

RETRACTED

Long non-coding RNAs (lncRNAs) are a critical group of non-protein coding RNA transcripts that have a length greater than 200 nucleotides. The main pathological changes of AS include proliferation, migration and apoptosis of vascular smooth muscle cells, etc. LncRNA plays a pivotal role in the regulation of these pathological processes. LncRNA HCG11 has a wide range of biological roles. HCG11 can affect the proliferation, invasion, metastasis and apoptosis of tumor cells [10–13]. However, the role of HCG11 in atherosclerosis is rarely reported. MicroRNAs (miRNAs) are about 20 to 25 nucleotides in size. Relevant experiments have confirmed that miRNAs play an important role in gene expression. MicroRNAs are involved in physiological and pathological processes such as ontogenesis, cell proliferation, differentiation, apoptosis, and atherosclerosis through targeted degradation of messenger RNA (mRNA) or inhibition of mRNA translation. Recent studies have confirmed that circulating miRNAs exist in a stable form in various body fluids, including plasma and urine, and can be used as biomarkers for diseases. Recent studies [14] have shown that miR-144 is not only an important regulator of erythrogenic differentiation, but also involved in the occurrence of diseases with high incidence rates such as tumors and cardiovascular and cerebrovascular diseases. About 50% of the identified lactation actin miRNAs exist in clusters in the genome and are transcribed as primary transcripts of polycistrons [15]. The precursor of miR-144 exists in the form of miR-144/miR-451 clusters.

FOXF1 is a class of transcription factors closely related to embryonic development and tumorigenesis [16]. Recent studies have found that FOXF1 gene plays an important regulatory role in gene expression in normal cells and tumor cells, and the abnormal expression of FOXF1 gene is closely related to the occurrence, progression and prognosis of various diseases [17–19]. FOXF1 gene can participate in the process of cell proliferation, invasion and metastasis through the expression of several genes and the regulation of different signaling pathways. At present, there are few reports on FOXF1 gene expression in AS and its role in AS [20–22].

RETRACTED

In this study, we aimed at exploring the expressions and functions of HCG11 in patients with AS. Firstly, we found that HCG11 was significantly increased in AS, which might contribute to the development of AS. Therefore, we wanted to investigate the functions and the underlying mechanism of HCG11 in AS patients.

## Methods

### Patient samples

Serum samples were collected from 20 AS patients and 20 healthy volunteers in the First Affiliated Hospital of Xi’an Jiaotong University from October 2018 to October 2019. There were no significant differences in age or sex between the patients and the healthy volunteers. All serum samples were frozen in liquid nitrogen at -80 °C. If the patient had other clinical diseases, the patient was excluded, and all the patients and healthy volunteers signed the informed consent. This study was approved by the ethics committee of the First Affiliated Hospital of Xi’an Jiaotong University and was in line with the principles of the Helsinki declaration.

### Cell culture

Human vascular smooth muscle cells (VSMCs) and HEK293 cells were purchased from American Type Culture Collection (ATCC, Manassas, VA, USA). The cells were routinely cultured in RPMI 1640 medium containing 10% Fetal Bovine Serum (FBS), 100 U/ml penicillin and 100 mg/ml streptomycin. The cells were grouped in predefined groups at 37 °C in a humidified incubator with 5% CO_2_.

### Cell transfection

The miR-144 mimics, miR-144 inhibitor and corresponding control (mimics NC and inhibitor NC) were all obtained from Shanghai GenePharma Co., Ltd. (Shanghai, China). The cDNA encoding HCG11 was amplified by PCR, and then ligated into pcDNA3.1 + vector (Invitrogen). Cell transfection was performed using Lipofectamine 2000 (Invitrogen). After 48 h, the transfection efficiency was validated by RT-qPCR analysis.

### AS animal model

High fat feed combined with vitamin D was used to prepare AS model. Wistar rats were randomly divided into 2 groups with 10 rats in each group. High-fat + vitamin D3 group: each group was intraperitoneally injected with vitamin D3 at a total amount of 700000U/kg, divided into 3 days. Subsequently, 20 g of high-fat feed (basal feed + 3.5% cholesterol +10% lard + 0.2% propylthiouracil + 0.5% sodium cholate +5% sugar) was given daily for 21 days. Control group: each rat was injected intraperitoneally with the same volume of normal saline every day, and given 20 g of standard feed after 3d, and fed continuously for 21d.

### CCK8 experiment

One day before the experiment, cells from different groups in the logarithmic growth stage were inoculated in 96-well plates, each well containing 1 × 10^3^ cells/well, and cultured in a 37 °C incubator for 72 h. Then, 10μL CCK-8 solution was added to each well and incubated in a 37 °C incubator for 2 h. Then, the photodensity (D) value of 450 nm was detected with an enzyme marker. The experiment was repeated three times.

RETRACTED

### Flow cytometry

After the cells were treated according to the requirements of each group, cells were digested and collected with trypsin, washed with precooled PBS at 4 °C for 2 times, then PBS was centrifuged, and the cells were resuspted with buffer solution. PI double fluorescence markers of 5μL Annexinv-FITC and 1μL 0.1 g/L were added, and apoptosis was detected by flow cytometry.

### TUNEL assay

Apoptosis was detected by TUNEL cell apoptosis detection kit. The cells were washed with PBS, fixed with 40 mL/L paraformaldehyde, and the cell membrane was penetrated with 1 mL/L TRitonX-100. Then the cells were washed with PBS, and the endogenous peroxides were inactivated with 3 mL/L H_2_O_2_. The biotin marker solution was configured according to the operating instructions for labeling reaction, and the color was developed with DAB and detected by fluorescence microscope.

### Qrt-pcr

The total RNA was extracted with TRIzol reagent (Invitrogen), and the concentration and purity of RNA were detected by NanoDrop before cDNA was synthesized. The reaction conditions were: denaturation at 40 °C for 60 min, 25 °C for 5 min, and 85 °C for 5 min. The expression levels of HCG11, miR-144-3p and FOXF1 were detected according to the instructions of the qPCR kit using cDNA as the template. The reaction conditions were: denaturation at 95 °C for 15 s, annealing at 55 °C for 30 s, extension at 72 °C for 10 s, and amplification of 30 cycles. Glyceraldehyde-3-phosphate dehydrogenase (GAPDH) was used as internal reference for HCG11 and FOXF1, and U6 was used as internal reference for miR-144-3p. The experiment was repeated for 3 times. The upstream primer of HCG11 is: 5′-uucuccgaacgugucacgutt-3′, and the downstream primer is: 5′-gccagaauguucauuatt-3′. The upstream primer of miR-144-3p was: 5′-cctcgcacctggaggctggctg-3’, and the downstream primer was: 5′-ttatcagttgggaaaatagta-3′. The upstream primer of GAPDH is: 5′-gtcaccttcaccgttccagtttttttt-3′, and the downstream primer is: 5′-cttagttgcgttacaccctttctt-3′. The upstream primer of U6 was: 5’-ctcgcttcggcagcacatatatact-3′, and the downstream primer was: 5′-acgcttcacgaatttgcgtgtc-3′. The primers were all synthesized by Kunming cycco biotechnology co., LTD. Each hole fluorescence signal reaches the threshold cycle number for experienced by Ct value, with 2^−ΔΔCt^ method to calculate the relative expression of the gene.

RETRACTED

### Double luciferase reporter assay

PCR was amplified to sequence fragments containing the binding sites of miR-144-3p to HCG11 and FOXF1 in the 3′UTR region, and imported into the pmirGLO luciferase expression vector to obtain the HCG11/FOXF1 wild-type vector (pmirGLO-HCG11-WT/pmirGLO-FOXF1-WT). The same method was used to obtain the HCG11/FOXF1 mutant vector (pmirGLO-HCG11-MUT/pmirGLO-FOXF1-MUT). PrirGLO, HCG11/FOXF1 wild-type vector, HCG11/FOXF1 mutant vector, miR-144-3p mimics and the negative control group were mixed with LipofectamineTM2000 liposomes and transfected with HEK293T and VSMCs cells, respectively. After transfection for 48 h, luciferase activity was detected according to the instructions of the dual-luciferase reporter gene detection kit.

### RNA pull down assay

When the cell fusion degree reached 90%, the cell scraper scraped off the cell, washed the scraper with 1 mL pre-cooled PBS, and the suspension was collected and placed in the EP tube. All the above operations were completed on ice. After centrifugation at 10000R/min at 4 °C for 30 s, cell precipitation was obtained, the supernatant was discarded, and 300 μL cell lysate (1.5 mg/mL heparin, 2 mmol/L DTT, protease inhibitor, and phosphatase inhibitor) was added to lyse cells at 4 °C for 1 h. The cells were centrifuged at 10000R/min at 4 °C for 10 min, and the lysed supernatant was collected into the DECP-treated EP tube without RNase enzyme. Biotin-labeled 3 ‘-UTR probes were added to the lytic supernatant for about 400 ng, yeast RNA (100 ng/mL, 1.5 μL), RNasein-hibitoR (0.1 U/μL, 3 μL), heparin (1.5 mg/mL), and incubated at 4 °C for 3 h. The 20 μL-labeled beads were placed in the RNase free EP tube, and the 500 μL-labeled beads were washed with the cell lysis fluid 500 μL. The beads were centrifuged at 4 °C for 5 min. The supernatant was discarded and set aside. After the probe was incubated with the lysate for 3 h, the beads were transferred to pre-washed beads after 10000R/min and centrifuged at 4 °C for 5 s. The beads were incubated at 4 °C for 3 h. After 3 h, the mixed solution was washed with 750 μL cell lysate to remove the non-specific proteins bound to the beads. The supernatant was discarded after centrifugation at 4 °C for 5 min. Repeat cleaning beads 4 times, then added 2 × Loading Buffer 20 μL 95 °C for 5 min, and centrifuge 11430R/min for 3 min for subsequent analysis.

### Statistical analysis

Using SPSS 19.0 software, all data are for repeat 3 times of experiments, measurement data in x ± s. Pearson linear correlation was used to analyze the correlation between LncRNA HCG11 and miR-144-3p expression. T test was used for comparison between two groups, and single factor ANOVA was used for comparison between multiple groups. P < 0.05 means the difference is statistically significant.

RETRACTED

## Results

The expression of HCG11 was up-regulated in patients with AS, and the expression of HCG11 was increased in ox-LDL and IL-6-induced VSMCs.

In order to explore the role of HCG11 in patients with AS, we first used qRT-PCR to detect the expression of HCG11 in the serum of patients with AS (n = 20) and healthy volunteers (n = 20). The results showed a significant increase in HCG11 in patients with AS compared to healthy volunteers (Fig. 1a). Furthermore, we used VSMCs as the cell model. VSMCs plays a key role in the development of AS. To evaluate the factors affecting the expression of HCG11 in VSMCs, we stimulated VSMCs with ox-LDL, IL-6, and TNFα, respectively. The experimental results showed that the expression of HCG11 was up-regulated after ox-LDL, IL-6 and TNFα stimulation (Fig. 1b–d). The above results showed that HCG11 was elevated in patients with AS, and ox-LDL, IL-6 and TNFα stimulation in VSMCs could up-regulate HCG11. We further constructed an animal model of atherosclerosis to detect the expression of HCG11 in the control group and the model group. Experimental results showed that HCG11 expression was up-regulated in the model group compared with the control group (Fig. 1e). The experimental results indicated that HCG11 may play a certain role in the process of AS disease.

**Fig. 1:** LncRNA HCG11 is up-regulated in AS patients and VSMCs cells induced by ox-LDL, IL-6 and TNFα. **a** HCG11 was upregulated in patients with AS. **b, c, d** Detection of HCG11 expression after different treatments. E. HCG11 was upregulated in AS model. *P < 0.5, **P < 0.01

### Overexpression of HCG11 promoted cell proliferation and inhibited apoptosis of VSMCs

In order to investigate the role of HCG11 in patients with AS, we constructed HCG11 overexpressed plasmids. After transfection of vector-NC and vector-HCG11 into VSMCs, the expression of HCG11 in the transfection group was significantly increased (Fig. 2a). The proliferation of VSMCs after transfection with HCG11 was evaluated by CCK8 method. The results showed that HCG11 overexpression increased the proliferation capacity of VSMCs compared with the blank control group and the NC group (Fig. 2b). Flow cytometry and TUNEL staining were used to detect apoptosis. The results showed that under the same induction of apoptosis, the apoptosis rate of the overexpressed HCG11 group was significantly lower than that of the other two groups (Fig. 2c, d). Further experimental results showed that after overexpression of HCG11, the protein level of anti-apoptotic gene Bcl-2 was increased, while the apoptotic gene Bax was significantly reduced (Fig. 2e, f). These results suggested that overexpression of HCG11 promoted cell proliferation and inhibited apoptosis of VSMCs.

RETRACTED

**Fig. 2:** HCG11 overexpression promotes cell proliferation and inhibits VSMCs apoptosis. **a**QPCR detection of HCG11 expression. **b** Cell proliferation assay. **c** Flow cytometry assay **d** TUNEL staining. **e, f** QPCR detection of Bax and Bal-2 expression. *P < 0.5, **P < 0.01. Magnification: 200 ×

### HCG11 directly targeted binding to miR-144

In order to further explore the potential mechanism of HCG11, we used StarBase v2.0 database to analyze the target cells and found that miR-144 was a potential target miRNA (Fig. 3a). Next, we carried out luciferase gene reporter gene experiment. The results showed that relative luciferase activity was significantly inhibited in VSMCs co-transfected with WT-HCG11 and miR-144 mimics, compared with cells transfected with mimics-NC. In cells co-transfected with MUT-HCG11, the results were reversed. In addition, similar results were found in HEK293 cells (Fig. 3b). Further, we confirmed through the HCG11 probe fishing experiment that HCG11 probe could significantly enrich miR-144 (Fig. 3c). In addition, the expression of miR-144 in VSMCs was significantly inhibited after transfection with HCG11 overexpression (Fig. 3d–e). We then measured the expression of miR-144 in patients with AS and healthy volunteers. The results showed that miR-144 was significantly reduced in patients with AS (n = 20) (Fig. 3f). In addition, the expression of miR-144 in VSMCs was inhibited after ox-LDL and IL-6 treatment (Fig. 3g, h). Further correlation test results showed that in patients with AS, miR-144 was negatively correlated with HCG11 (Fig. 3i). These results suggest that HCG11 can directly bind to miR-144 in VSMCs, possibly as a ceRNA regulating the development of AS.

**Fig. 3:** HCG11 directly binds to miR-144-3p. **a** Binding site of HCG11 and miR-144. **b** Dual luciferase reporter gene assay. **c** RNA pull down experiment. **d** Transfection efficiency verification. **e** Detection of miR-144 expression. **f** MiR-144 is down-regulated in AS patients. **g** Detection of miR-144 expression in VSMCs. **h** Detection of miR-144 expression. **i** Detection of the coexpression of HCG11 and miR-144. *P < 0.5, **P < 0.01

### MiR-144 inhibited the proliferation of VSMCs and promotes apoptosis

To further investigate the potential role of miR-144 in patients with AS, miR-144 mimic or mimics-NC were transfected into VSMCs, respectively. The results showed that miR-144 mimics could significantly up-regulate the expression of miR-144 (Fig. 4a). The proliferation capacity of VSMCs cells transfected with miR-144 mimics was significantly reduced (Fig. 4b). Apoptosis was significantly increased after overexpression of miR-144 (Fig. 4c, d). After overexpression of miR-144, the protein level of Bcl-2 decreased and the level of apoptotic gene Bax increased (Fig. 4e, f). Together, these results revealed that miR-144 overexpression inhibited VSMCs cell proliferation and promoted VSMCs cell apoptosis. However, the specific mechanism of miR-144 in AS remains to be further studied.

RETRACTED

**Fig. 4:** MiR-144 inhibits the proliferation of VSMCs and promotes apoptosis. **a** The expression of miR-144 in VSMCs after different treatment. **b** Cell proliferation assay. **c** Flow cytometry assay. **d** TUNEL staining. **e, f** QPCR detection of Bax and Bcl-2 expression. *P < 0.5, **P < 0.01. Magnification: 200 ×

### MiR-144 targeted and binded to FOXF1 in VSMCs

In order to further explore the mechanism of miR-144 inhibiting VSMCs cell proliferation and promoting apoptosis. We used the TargetScan database to predict the target genes of miR-144. FOXF1 was predicted as a target gene for miR-144 (Fig. 5a). Next, we performed luciferase gene reporter gene test for validation. The results showed that the relative luciferase activity was inhibited in the VSMCs co-transfected with the WT-FOXF1 and miR-144 mimics, while the relative luciferase activity remained unchanged in the cells co-transfected with the MUT-FOXF1 and miR-144 mimics. In addition, similar results were found in HEK293 cells (Fig. 5b). The enrichment analysis results also showed that miR-144 probe could be significantly enriched to FOXF1 (Fig. 5c). Further experimental results showed that FOXF1 protein levels were significantly inhibited in the miR-144 stimulation group compared with the control group, and FOXF1 expression was up-regulated after miR-144 inhibition (Fig. 5d, e). In addition, FOXF1 expression in VSMCs was up-regulated after ox-LDL treatment (Fig. 5f). These data suggest that in VSMCs, miR-144 can be directly targeted to bind to FOXF1. We analyzed the coexpression correlation between HCG11 and FOXF1 in AS patient tissues. The experimental results showed that HCG11 was positively correlated with FOXF1 co-expression (Fig. 5g, R square = 0.4596, P = 0.0312).

**Fig. 5:** MiR-144 binds to FOXF1 in VSMCs. **a** Binding site of FOXF1 and miR-144. **b** Dual luciferase reporter gene assay. **c** RNA pull down experiments. **d** Verification of transfection efficiency. **e, f** Detection of FOXF1 expression. G. Co-expression correlation between HCG11 and FOXF1 in AS patient tissues. *P < 0.5, **P < 0.01

RETRACTED

### HCG11 promoted cell proliferation and inhibited apoptosis in VSMCs through miR-144/FOXF1

To further validate the hypothesis, we transfected miR-144 mimic or HCG11 into VSMCs. The results showed that the expression of FOXF1 was up-regulated after the overexpression of HCG11. After transfection with miR-144, FOXF1 expression was down-regulated. However, miR-144 mimics could reverse the effect of HCG11 (Fig. 6a). CCK8 showed that the proliferation of HCG11 cells was enhanced after overexpression, while the proliferation of miR-144 cells was inhibited after simulated transfection. Moreover, miR-144 mimics could reverse the effect of HCG11 (Fig. 6b). The results of flow cytometry and TUNEL staining showed that the apoptosis rate decreased after overexpression of HCG11, while increased after overexpression of miR-144 (Fig. 6c, d). In addition, after overexpression of HCG11, the Bcl-2 protein level increased and Bax level decreased, while the reverse was observed after transfection of miR-144 (Fig. 6e, f). In summary, our study found that HCG11 was upregulated in AS samples, which may be spongy with miR-144, while inhibited miR-144 can increase the expression of FOXF1, thus promoting the proliferation of VSMCs and regulating the development of AS.

**Fig. 6:** HCG11 promotes cell proliferation and inhibits apoptosis in VSMCs through miR-144/FOXF1. **a** Detection of FOXF1 expression. **b** Cell proliferation assay. **c** Flow Cytometry assay. **d** TUNEL staining. **e** QPCR detection of Bax and Bcl-2 expression. *P < 0.5, **P < 0.01. Magnification: 200 ×

## Discussion

With the improvement of people’s living conditions, the incidence of arterial vascular diseases is increasing year by year. AS is the main manifestation of vascular diseases, and also the common pathological basis of coronary heart disease and cerebrovascular diseases, which have serious harm to people’s health [23, 24]. The substance of AS is a chronic vascular inflammatory disease characterized by lipid deposition in the tube wall, mainly manifested AS endothelial dysfunction, formation of foam cells and proliferation of smooth muscle cells, etc. [25–27]. Vascular smooth muscle cells (VSMCs) are one of the main cells that constitute the structure of vascular wall tissue and maintain vascular tension. The structural and functional changes of VSMCs are the cytopathological basis of various cardiovascular diseases such as hypertension, atherosclerosis and restenosis after angioplasty [28, 29]. The purpose of this study was to describe the regulatory role of the HCG11/miR-144/FOXF1 axis in AS and to describe the cellular/molecular mechanisms of this axis function.

RETRACTED

A series of recent studies have found that transcription related to the pathogenesis of atherosclerotic plaques [30], hypoxia-inducible factor 1 leux-antisense RNA1 [31], MIAT [32], SENCR [33] and other relevant genes play a crucial role in the proliferation and apoptosis of vascular smooth muscle cells. LncRNAs are a new class of cell proliferation and apoptosis regulators and can also be used as therapeutic targets for atherosclerosis and related cardiovascular diseases. Through RNA sequencing, Ballantyne et al. [34] found a new lncRNA named SMILR. After conditioned stimulation, the expression of SMILR in both the nucleus and cytoplasm increased, while the degradation of SMILR significantly reduced the proliferation of smooth muscle cells. In human blood samples, they also observed increased expression of SMILR in unstable AS plaques and elevated plasma c-reactive protein levels, suggesting that SMILR may be a driver of proliferation of VSMCs. Li et al. [35] found that, compared with normal vascular tissue, the expression level of lncRNA BANCR in the AS plaque tissue was up-regulated, and in the proliferating VSMCs, BANCR regulated the proliferation and migration of VSMCs by activating the JNK pathway. Taking lncRNA AS the target, the mechanism of lncRNA regulating the proliferation and differentiation function of VSMCs was further studied, so AS to inhibit the abnormal proliferation of VSMCs and keep it in the dynamic equilibrium process, which helped to delay the process of AS. This is expected to be a new strategy to reduce AS and other lesions. Our experiment yielded several new discoveries. We found that HCG11 was negatively correlated with miR-144 expression, with the former up-regulated in AS and the latter down-regulated. In addition, overexpression of HCG11 significantly promoted the progression of AS disease.

The researchers found that microRNAs play an important role in the cardiovascular physiological and pathological process, it can be applied to a variety of genetic regulation of cardiovascular disease, research shows that the miRNA can be adjusted by the expression of intercellular adhesion molecules and inflammatory factor, the process of cell cycle and cell proliferation, lipid metabolism, the function of endothelial cells and angiogenesis, plaque formation and rupture and directly or indirectly participate in the regulation of vascular endothelial cells, vascular smooth muscle cells and the function of macrophages, which affect the AS and pathophysiological process of cardiovascular disease [36]. Ovcharenko et al. [37] demonstrated that the introduction of miRNAs such as let-7c and miR-144 could affect the Caspase cascade reaction activity, and the predicted targets of these endogenous miRNAs included the encoding of death receptors, Caspases and other genes related to apoptosis. Transfection of miR-144 analogues into rat H9C2 cardiac myocytes showed a significant decrease in cell proliferation, a significant increase in caspase-3 activity, and a significant increase in apoptosis rate [38], suggesting that miR-144 is a gene promoting apoptosis of cardiac myocytes. MiR-144/451 provides a new target for the treatment of ischemic heart disease and congenital heart disease. FOXF1, as an important forkhead transcription factor, is usually expressed in mesenchymal cells and promotes the transfer of mesenchymal cells by increasing the movement of fibers [19, 22]. FOXF1 plays an important role in regulating the expression of multiple genes and different signaling pathways. FOXF1, as the target gene of miR-144, may mediate the pro-proliferation and pro-apoptotic effects of the HCG11/miR-144 axis. In this study, it was found that FOXF1, AS a target gene of miR-144, may mediate the promotion effect of AS on the HCG11/miR-144 axis. HCG11 limits the functional availability of miR-144 through sequence complementation as ceRNA. Therefore, our study reveals new aspects of the cellular function and pathophysiological role of HCG11 and miR-144, both of which can be considered AS potential molecular targets for the treatment of AS. The shortcoming of this study is that there is no further study on the downstream molecular mechanism of FOXF1.

RETRACTED

## Conclusions

We found that HCG11 was upregulated in AS patients. Furthermore, HCG11 overexpression promoted cell proliferation and inhibited cell apoptosis via targeting miR-144/FOXF1 signaling axis. Our results elucidated a potential mechanism underlying the role of HCG11, which might be used as a promising marker and a potential target for AS patients.

## Data Availability

The datasets used and/or analyzed during the current study are available from the corresponding author on reasonable request.

## Abbreviations

AS: Atherosclerosis
lncRNA: Long non-coding RNA
QRT-PCR: Quantitative real-time polymerase chain reaction
Ox-LDL: Oxidation low lipoprotein
IL-6: Interleukin-6
TNF α: Tumor necrosis factor α
VSMCs: Vascular smooth muscle cells
FOXF1: Forkhead box protein F1
Bcl-2: B-cell lymphoma-2
Bax: BCL2-Associated X
CCK-8 assay: Cell Counting Kit-8 assay
TUNEL staining: Terminal deoxynucleotidyl transferase-mediated dUTP-biotin nick end labeling assay staining
GAPDH: Glyceraldehyde-3-phosphate dehydrogenase
